The article "Efficacy Evaluation of Inflammatory Mediators in the Treatment of Multiple Myeloma with Daratumumab" was retracted in 2023. Reasons: signs of a paper mill; suspected computer-generated content; unreliable results or conclusions; lack of ethics approval or compliance.

# Efficacy Evaluation of Inflammatory Mediators in the Treatment of Multiple Myeloma with Daratumumab

**DOI:** 10.1155/2022/9350211

**Published:** 2022-08-27

**Authors:** Jie Meng, Xiaoyu Zhao, Duanfeng Jiang, Changjiu Liang, Xunxiu Ji, Min Dong

**Affiliations:** ^1^The Second Affiliated Hospital of Hainan Medical University, Haikou 570216, Hainan, China; ^2^Institute of Microbiology, Heilongjiang Academy of Sciences, Harbin 150010, Heilongjiang, China

## Abstract

**Objective:**

This study aimed to investigate the regulatory ability and clinical therapeutic effect of daratumumab on inflammatory mediators in patients with multiple myeloma.

**Method:**

The Multiple Myeloma Public Genetic Data Array download GSE125361 dataset was collected. The GO analysis and KEGG analysis were performed on the differential genes to elucidate the multiple myeloma cytokine-related gene pathways. Daratumumab is a CD38 monoclonal antibody used to treat multiple myeloma. Patients with newly diagnosed multiple myeloma were treated with monoclonal antibodies containing CD38, and the control group was treated with a regimen without daratumumab. The serum levels of IL-2, IL-4, IL-6, IL-10, TNF-*α*, and IFN-*γ* were measured in the two groups before and after treatment and the therapeutic effects of the two groups were compared.

**Result:**

The KEGG analysis showed that the Th17 cell differentiation, apoptosis, and cytokine-cytokine receptor interaction pathways were differentially expressed in multiple myeloma. The expression levels of serum IL-2, IL-6, IL-10, and TNF-*α* in patients in the daratumumab group were lower than those in the control group after chemotherapy. The overall effective rate of patients treated with daratumumab after chemotherapy was higher than that of the control group.

**Conclusion:**

Daratumumab can effectively improve the levels of IL-2, IL-6, IL-10, and TNF-*α* in patients with multiple myeloma and improve the therapeutic effect.

## 1. Introduction

Multiple myeloma (MM) is a malignant proliferative disease caused by the abnormal production of B cell monoclonal M protein [1–4]. Clinically, MM is accompanied by complications such as osteolytic injury, repeated infection, and kidney injury [5]. Epidemiological statistics demonstrated that multiple myeloma has a high incidence rate, and it has become the second hematological malignancy after leukemia and lymphoma [6]. Myeloma cells can enter the bone marrow through interactions with stromal cells and osteoblasts, which in turn affect the generation of plasma cells and the differentiation of myeloma cells [7]. The involvement of inflammatory mediators is essential and IL-6 can promote the growth of multiple myeloma cells [8]. Inflammatory pathways such as NF-*κ*B can also promote the growth of multiple myeloma [9]. With the development of pharmacological research, the CD38 monoclonal antibody for the treatment of multiple myeloma, namely, daratumumab, has made a qualitative leap in the efficacy of multiple myeloma treatment. Daratumumab is a humanized, antiCD38 IgG1 monoclonal antibody that binds to CD38 expressed by tumor cells through complement-dependent cytotoxicity (CDC), antibody-dependent cell-mediated cytotoxicity (ADCC), and antibody-dependent phagocytosis (ADCP), as well as Fc*γ* receptors and other immune-related mechanisms, to induce tumor cell apoptosis [10]. The current research study on this drug is limited to the complement pathway, antibody-dependent pathway, phagocytosis, and so on. The effect of daratumumab on inflammatory mediators has not been established. The guiding significance of inflammatory mediators in the judgment of clinical efficacy is not yet clear. In this experiment, the method of bioinformatics research will be used to mine inflammatory mediator-related genes in multiple myeloma, and then, the ELISA method will be used to detect the level of inflammatory mediators in serum, and the clinical treatment effect will be calculated. This study will provide some experience for the clinical treatment of multiple myeloma with daratumumab.

The article "Efficacy Evaluation of Inflammatory Mediators in the Treatment of Multiple Myeloma with Daratumumab" was retracted in 2023. Reasons: signs of a paper mill; suspected computer-generated content; unreliable results or conclusions; lack of ethics approval or compliance.

## 2. Materials and Methods

### 2.1. Data Collection

The genetic data involved in this study are the GSE125361 chip carried in the public gene chip data platform database on the website of the American National Center for Biotechnology Information, and the chip platform is GPL20844 Agilent-072363 SurePrint G3 Human GE v3 8 × 60 K Microarray 039494. This version contains mRNA from 45 multiple myeloma samples and 3 control tissue mRNAs.

### 2.2. Screening of Differential Genes

The analysis of the downloaded data chip was carried out by the R program, which read all the matrix files and then analyzed the multiple myeloma tissue data set and the control group tissue data set with the LIMMA function analysis package to obtain the differentially expressed genes, and then deduplicate the data results. The threshold for filtering was set as log2FC ≥ 1 or log2FC ≤ −1, absolute value<0.05. Then, the GGPLOT function package was used to load the R program and draw the volcano map.

### 2.3. Patient Data

A total of 21 patients with multiple myeloma who were admitted to the First District of the Hematology and Cell Therapy Department of the Second Affiliated Hospital of Hainan Medical University between June 2020 and April 2022 were selected. The patients included 9 males and 12 females, aged 51–86 years, with an average age of 67 years. The inclusion criteria for this study were clinical symptoms and auxiliary examinations of the patients. They all met the relevant requirements of the Chinese Guidelines for the Diagnosis and Treatment of Multiple Myeloma. The exclusion criteria were as follows: (1) The patient had a history of infection. (2) The patient is missing, lost to follow-up, or died. (3) The patient's family refused to sign the informed consent. (4) Patients with organ failure. (5) Patients with an impaired liver and kidney function.

The article "Efficacy Evaluation of Inflammatory Mediators in the Treatment of Multiple Myeloma with Daratumumab" was retracted in 2023. Reasons: signs of a paper mill; suspected computer-generated content; unreliable results or conclusions; lack of ethics approval or compliance.

### 2.4. Grouping

Patients were grouped according to whether they were treated with daratumumab. There were 7 males and 7 females in the control group (without daratumumab), aged 51–82 years, with an average age of 68 years. In the experimental group (using daratumumab), there were 2 males and 5 females, aged 52–81 years, with an average age of 65 years. On the basis of the control group, oral administration of daratumumab was added to the experimental group.

### 2.5. Detection of Serum Cytokines

The nursing staff used a vacuum anticoagulation tube coated with EDTA to collect 5 ml of cubital venous blood for all patients after admission, before chemotherapy, and after each chemotherapy for the first ten times. After the collection, the samples of the patients were sent to the laboratory for examination. The levels of IL-2, IL-4, IL-6, IL-10, TNF-*α*, and IFN-*γ* were measured using commercial ELISA kits (Beyotime, China) according to the manufacturer's instructions.

### 2.6. Patient Evaluation

The efficacy evaluation indexes of patients involved blood routine, liver function, renal function, serum ions, immunoglobulin, *β*-microglobulin, bone marrow image, and protein electrophoresis.

### 2.7. Statistical Analysis

The statistical analysis was performed using SPSS 24.0 software (IBM SPSS Statistics, Chicago, USA). The data were presented as mean ± standard deviation (SD). All data were first tested for homogeneity of variance. After the homogeneity of variance test was satisfied, the *T* test was used for the measurement data and the chi-squared test was used for the count data. Differences within groups were analyzed by the *F* test and sequence data by the Wilcox-rank sum test. A two-sided *P* value less than 0.05 was considered statistically significant.

## 3. Result

### 3.1. The Differential Gene Expression of the GSE125361 Dataset

As shown in Figures 1(a) and 1(b), a total of 3553 differential genes, of which 1430 were upregulated and 2123 were downregulated, were identified in the GSE125361 dataset. In the volcano map, the genes with FC differences more than 2 times and statistically significant differences were counted and observed. The GO analysis of upregulated genes revealed biological processes focused on endoplasmic reticulum unfolded protein response, ubiquitin-dependent ERAD pathway, response to endoplasmic reticulum stress, apoptotic processes, negative regulation of viral processes, cellular components involved in membrane components of the receptor complex, components of the endoplasmic reticulum membrane, endoplasmic reticulum membrane, and endoplasmic reticulum. The KEGG-involved pathway includes protein processing in the endoplasmic reticulum, Th17 cell differentiation, apoptosis, and cytokine-cytokine receptor interaction.

The article "Efficacy Evaluation of Inflammatory Mediators in the Treatment of Multiple Myeloma with Daratumumab" was retracted in 2023. Reasons: signs of a paper mill; suspected computer-generated content; unreliable results or conclusions; lack of ethics approval or compliance.

### 3.2. GO and KEGG Analysis of Differential Genes

GO and KEGG signaling pathway enrichment analysis of upregulated genes was performed using David's website online analysis of differential genes, and the specific results are shown in Figure 2. The GO analysis showed that biological processes were concentrated in the endoplasmic reticulum unfolded protein response, ubiquitin-dependent ERAD pathway, response to endoplasmic reticulum stress, apoptosis process, negative regulation of the viral process, cellular components involved in membrane components, receptor complex, components of endoplasmic reticulum membrane, endoplasmic reticulum membrane, and endoplasmic reticulum. The KEGG-involved pathway included protein processing in the endoplasmic reticulum, Th17 cell differentiation, apoptosis, and cytokine-cytokine receptor interaction. The genes involved in cytokine-cytokine receptor interactions include TNFRSF17, BMP4, BMP6, BMPR1A, CD40, CCR10, IFNAR2, IL2RB, IL5RA, IL6R, IL6ST, IL12RB1, IL15, IL16, CCL3, CCL24, XCL1, TNFRSF14, TNFRSF10A, IL32, IL27RA, CCL4L2, TNFRSF13B, IL22RA1, EDA2R, ACVR1C, IFNLR1, and BMP8A (see Figure 3).

### 3.3. Basic Information of Patients in the Two Groups

The basic data of patients in the two groups are shown in Table 1. The statistical analysis of the basic data of the patients in the daratumumab group compared with the control group showed that the data difference was not statistically significant (*P* > 0.05).

### 3.4. Serum Levels of Inflammatory Cytokines in the Two Groups of Patients

The expression levels of serum inflammatory factors in the two groups of patients are shown in Table 2. The serum levels of IL-2, IL-6, IL-10, and TNF-*α* in patients in the daratumumab group were significantly lower than those in the control group (*P* < 0.05).

### 3.5. Curative Effect Distribution of Patients in the Two Groups

The therapeutic effects of the two groups are shown in Table 3. The treatment effect in the daratumumab group was significantly higher than that in the control group (*P* < 0.05).

The article "Efficacy Evaluation of Inflammatory Mediators in the Treatment of Multiple Myeloma with Daratumumab" was retracted in 2023. Reasons: signs of a paper mill; suspected computer-generated content; unreliable results or conclusions; lack of ethics approval or compliance.

## 4. Discussion

Multiple myeloma is the most common malignant plasma cell tumor, and abnormal serum cytokines are the most common phenomena in patients with multiple myeloma. At present, the cause of abnormal serum cytokines is not clear, but it is generally believed that these inflammatory factors are autocrine by tumor cells or secreted by lymphocytes after tumor stimulation. Several growth factors have been shown to promote the growth of multiple myeloma tumors. In this study, the activation of the cytokine-cytokine receptor interaction pathway was found to be an obvious KEGG pathway in differentially expressed genes by selecting microarray data sets from multiple myeloma tissues. TNFRSF17, BMP4, BMP6, BMPR1A, CD40, CCR10, IFNAR2, IL2RB, IL5RA, IL6R, IL6ST, IL12RB1, IL15, IL16, CCL3, CCL24, XCL1, TNFRSF14, TNFRSF10A, IL32, IL27RA, CCL4L2, TNFRSF13B, IL22RA1, EDA2R, ACVR1C, IFNLR1, and BMP8A are genes activated in this pathway. Among them, TNFRSF14 and TNFRSF10A are the code genes of TNF receptor family member proteins, IL6R and IL6ST are the code genes of IL-6 receptor proteins, IL2RB is the code gene of the IL-2 receptor protein family, and IFNLR1 is the code gene of the IL-10 receptor protein. The activation of these genes indicates that the translation level of the receptor protein has increased, and the reason for the upregulation of the receptor is the increase in the number of ligands. IL-6, IL-2, IL-10, and TNF-*α* play a prominent role in the pathogenesis of multiple myeloma.

IL-6 is an important cytokine for multiple myeloma cell growth [11–14], which can be secreted by bone marrow stromal cells. IL-6R is a transmembrane protein on the cell membrane, and its binding to IL-6 triggers the activation of the Jak-STAT pathway [15], leading to further gene activation. At the same time, IL-6 can also promote cell proliferation directly through the activation of the RAS-MAP pathway [16]. IL-10 promotes cell proliferation by inducing the expression of IL-11 [17]. IL-2 and TNF-*α* are cytokines that play a protective role in multiple myeloma [18]. TNF-*α* is an important molecule in the autoimmune stage of the body, which has a certain role in tumor killing and inhibiting tumor growth [19]. IL-2 can induce the production of NK cells and increase the ability to dissolve tumor cells [20]. The data in Table 2 show that the levels of IL-2 and TNF-*α* are lower in patients treated with daratumumab in this experiment. This may be due to the toxic effects of the drug on multiple myeloma cells, which cause cell damage, and the decrease in cell numbers reduces the body's related mechanism of killing it. The decrease of IL-6 and IL-10 indicates that when daratumumab is used in the treatment of multiple myeloma, its main mechanism of tumor inhibition is related to it. Daratumumab is a monoclonal antibody drug against CD38. This drug can induce cytolytic death through the interaction of cytotoxicity, antibody-dependent cellular cytotoxicity, and antibody-dependent cellular phagocytosis. This drug can also adjust the immune microenvironment of tumors and eliminate the inhibitory ability of TREGS, BREGS, and other cells, to improve the level of inflammatory factors. In this experiment, through the data in Table 3, it can be found that daratumumab is more effective in patients. The reason for this phenomenon is not only that the drug can kill myeloma but also that the drug can increase the secretion level of the myeloma stroma and cytokines. Therefore, improving the cytokines of the tumor microenvironment is an important mechanism to improve the treatment of multiple myeloma.

The article "Efficacy Evaluation of Inflammatory Mediators in the Treatment of Multiple Myeloma with Daratumumab" was retracted in 2023. Reasons: signs of a paper mill; suspected computer-generated content; unreliable results or conclusions; lack of ethics approval or compliance.

In conclusion, daratumumab can inhibit the expression levels of IL-6, IL-2, IL-10, and TNF-*α* in patients with multiple myeloma, thereby inhibiting the growth of multiple myeloma. However, this experiment cannot carry out the verification of related genes due to the limitation of conditions. In future research, we will verify the expression level of related genes by the RT-qPCR method, in order to expect to obtain more abundant theoretical results.

## Figures and Tables

**Figure 1:** (a) Expression heat map of the dataset and (b) volcano plots showing differentially expressed genes.

**Figure 2:** (a) GO and (b, c, d) KEGG pathway enrichment of dataset.

**Figure 3:** (a) KEGG. (b) KEGG. (c) BP. and (d) CC.

**Table 1:** Disease characteristics of enrolled patients.

	Experimental group	Control group
Gender	2 : 5	7 : 7
Age	Age 52–81 (average 65)	Age 51–82 (average 68)
DS staging ratio (I : II : III)	0 : 0 : 100%	0 : 0 : 100%
ISS staging ratio (I : II : III)	1 : 4:2	1 : 5 : 8
R-ISS staging ratio (I : II : III)	0 : 1:6	1 : 6 : 7
SMART staging (standard risk: high risk)	1 : 6	10 : 4

**Table 2:** Serum levels of inflammatory factors in the two groups.

	IL-2	IL-4	IL-6	IL-10	TNF-*α*	INF-*γ*
Experimental group (pg/ml)	62.53	0.52	489.34	72.69	3.36	17.12
Control group (pg/ml)	<0.97	0.57	10.58	1.75	<0.85	16.15

**Table 3:** Curative effect of patients in the two groups.

	Complete remission (%)	Very good partial remission. (%)	Partial remission (%)	Ineffective (%)
Experimental group	14.29	42.86	28.57	14.29
Control group	0	33.33	55.56	11.11

## Data Availability

All the data are within the manuscript.
